The article "Construction of English Translation Model Based on Neural Network Fuzzy Semantic Optimal Control" was published in 2022. Journal: Comput Intell Neurosci.

# Construction of English Translation Model Based on Neural Network Fuzzy Semantic Optimal Control

**DOI:** 10.1155/2022/9308236

**Published:** 2022-05-02

**Authors:** Bingjie Zhang, Yiming Liu

**Affiliations:** ^1^School of English Language and Culture, Xi'an Fanyi University, Xi'an, Shaanxi 710105, China; ^2^School of Foreign Languages, Xidian University, Xi'an, Shaanxi 710126, China

## Abstract

This work addresses four aspects of the English translation model: consistency, model structure, semantic understanding, and knowledge fusion. To solve the problem of lack of personality consistency in the responses generated by neural networks in English translation models, an English translation model with fuzzy semantic optimal control of neural networks is proposed in this study. The model uses a fuzzy semantic optimal control retrieval mechanism to obtain appropriate information from an externally set English information table; to further improve the effectiveness of the model in retrieving correct information, this work adopts a two-stage training method, using ordinary English translation data for model pretraining and then fine-tuning the model using English translation data with optimal control containing fuzzy semantic information. The model consists of two parts, a sequence generation network that can output the probability distribution of words and an evaluation network that can predict future whole-sentence returns. In particular, the evaluation network can evaluate the impact of currently generated words on whole sentences using deep inheritance features so that the model can consider not only the optimal solution for the current words, as in other generative models, but also the optimal solution for future generated whole sentences. The experimental results show that the English translation model with fuzzy semantic optimal control of the neural network proposed in this study can obtain better semantic feature representation by using a novel bidirectional neural network and a masked language model to train sentence vectors; the combination of semantic features and fuzzy semantic similarity features can obtain higher scoring accuracy and better model generalization. In English translation applications, there are large improvements in scoring accuracy and generality.

## 1. Introduction

With the development of artificial intelligence and the wide application of deep learning technology in natural language processing (especially neural machine translation), the performance of machine translation is becoming more and more powerful. However, for the time being, most of the research in domestic academia and practice in the industry use English as the source language and English language for machine translation, and the research on translation between English and other languages is still far from enough [1, 2]. Under the situation of economic globalization and integration, economic, trade, and cultural exchanges are rapidly increasing, and the research on Chinese-French neural machine translation can help to further strengthen the exchanges between the two countries. However, since English has incomplete equivalence in lexical and syntactic aspects, no matching, and variation in verb tense and person, such incomplete equivalence undoubtedly brings greater difficulties and challenges to neural machine translation [3]. For English translation tasks, they can be classified into different levels according to different categorization methods. According to the granularity of processed text, it can be classified into word level, sentence level, and chapter level. According to the research methods, they can be classified as supervised learning, semisupervised learning, and unsupervised learning. Traditional classification algorithms mainly use manually constructed feature selection methods to perform feature extraction and train classifiers to finally complete the classification task. The performance of these classification methods heavily relies on the extraction of text features [4]. The description and modeling of nonlinear systems have become a hot research issue. Neural network fuzzy semantic optimization control technology has quickly become the key research object of experts and scholars due to its strong fitting ability and excellent characteristics of universal approximation. Many translation algorithms based on neural network fuzzy semantic optimization control technology have been proposed. In the translation system, the use of mathematical tools such as neural network fuzzy semantic optimization control technology to further accurately describe the motion state of the maneuvering target still has very important research value [5].

The article "Construction of English Translation Model Based on Neural Network Fuzzy Semantic Optimal Control" was published in 2022. Journal: Comput Intell Neurosci.

Since English translation models have very promising applications, they have been rapidly developed in both academic and industrial circles. At present, before the emergence of deep learning technology, the traditional research ideas are mainly divided into two types: linguistic rule/template-based approach and retrieval-based approach. However, researchers have found that with the increasing complexity of application scenarios and the increasing user requirements for interaction experience, rule-based matching approaches cannot meet these needs [6, 7]. While retrieval-based chatbots can ensure the grammatical rationality and fluency of the replies, they are limited by the richness of the training data, and the English translation model cannot give more satisfactory responses if the user's required replies are not in the conversation database. Deep learning techniques can solve the problems that are difficult to solve by traditional methods in English translation models and enable robots to learn dialogue patterns from a large amount of dialogue data so that they can effectively respond to any input from users. However, the existing deep learning methods still have defects such as poor response quality, inconsistent responses, and errors in semantic understanding, which are to be further explored in depth, which is also the significance of this research [8]. Deep learning methods can transform the text into vector representation for deep semantic extraction. Two-way long- and short-term memory networks can memorize the input information above and combine the data information above to influence the output of the later text and represent the contextual information of the text to extract the features of utterance sequences and semantics. Combining the deep semantic and shallow linguistic features, the constructed model can solve the automatic scoring problem of the English translation by combining fuzzy semantics and text fuzzy semantic similarity to calculate a reasonable score [9].

This study presents a neural network fuzzy semantic optimal control model for English translation. The model uses inherited features to unify the data and English for the training and testing process and gives the model the ability to focus on whole-sentence generation. The proposed model takes into account the rubric of the task and the long-term payoff of model decoding and is trained and tested on a large-scale English translation corpus, demonstrating significant enhancement effects [10]. In the first chapter, the research background, significance of this topic, and the main research content of this study are introduced. Chapter 2, related work, briefly analyzes the scoring problem of English translation model. The existing text fuzzy semantic similarity algorithm, word vector and sentence vector representation methods, and English translation model based on neural network fuzzy semantic optimal control are investigated. In the third chapter, the English translation score points and basis are analyzed, and then, the candidate features are summarized and extracted, including shallow linguistic features: lexical features (lexical number ratio, named entities, and keywords), sentence features, and deep semantic features, combined with fuzzy semantic similarity, and finally, the English translation model is constructed. The combination of semantic features and fuzzy semantic similarity features makes the scoring more accurate and has better generalizability. In chapter 4, the results are analyzed to compare different algorithmic models using two datasets, and after experiments on English translation-related datasets, the accuracy and efficiency of the proposed model on knowledge decision and response generation tasks are demonstrated. Chapter 5 is as follows: summary and prospect. The research work covered in this study is summarized and concluded; then, the shortcomings of this study and the current problems that still need to be solved are presented, and finally, the future research trends have prospected.

The article "Construction of English Translation Model Based on Neural Network Fuzzy Semantic Optimal Control" was published in 2022. Journal: Comput Intell Neurosci.

### 1.1. Related Research

Deep learning can automatically extract features from the text by building neural networks, without the need to manually design features. The principle is that deep semantic features of the text are learned and then classified by classifiers [11]. With the development of deep learning theory and word vector technology, neural network models have been gradually applied to English translation tasks and are favored by many scholars. Madani et al. used CNN to model sentences and completed English translation tasks on this basis with better results than traditional methods and achieved good results on several datasets [12]. Reyes-Magaña et al. proposed the Tree-LSTM model for predicting the semantic relevance of text and English translation,which is used to predictthe semantic relevance of text and English classification [13]. In recent years, the Attention model in deep learning was first used for machine translation by Yuan Z et al. Later, various variants of the Attention model were also applied to English translation work [14]. Chen et al. proposed a multiattentional convolutional neural network and used it for English classification of specific English, which can obtain deeper information on English features and effectively identify the English polarity of different English languages [15]. Neural network English translation has entered the field of vision of more and more people, providing convenient and fast translation services for more and more users, and has become an indispensable part of the public's daily life and communication. However, due to the explosive growth of multilingual information, people's demand for translation between different languages has increased, and there are higher requirements for the accuracy, fluency, and speed of neural network English translation [16]. One of the key reasons for the gap between human translation and human translation is the lack of rich translation knowledge of various granularities. For the research of neural network English translation, the research results of other languages can be used for reference in the research process.

The article "Construction of English Translation Model Based on Neural Network Fuzzy Semantic Optimal Control" was published in 2022. Journal: Comput Intell Neurosci.

With the rapid development of technology and continuous acceleration of the economic process, machine translation has become an important link of international cooperation and exchange [17]. With the development of artificial intelligence, the addition of deep learning technologies such as RNN and LSTM has changed the pattern of traditional machine translation in China, and the machine translation technology has been further developed in the new era, and the biggest change is the transformation from PBMT to NMT, which undoubtedly promotes the rapid improvement of machine translation quality. Chen et al. used multitask learning and semisupervised learning to improve the translation performance of NMT on resource-scarce languages [18]. Alom et al. used the method of incorporating bilingual dictionaries and linguistic knowledge to incorporate external prior knowledge into neural machine translation, a study on a fuzzy semantic-based approach to modeling NMT decoders. They also applied fuzzy semantic knowledge to NMT and also included a fuzzy semantic-level decoder and word-level decoder, similar to AI Lab's approach [19]. The main feature of the fuzzy model is to use multiple linear systems to deconstruct the input quantity through some methods in fuzzy mathematics and then defuzzy through fuzzy reasoning, thereby generating multiple sets of linear input and output functions, so as to solve complex nonlinear problems. The system is fitted [20].

In this study, we analyze the English translation scoring criteria, and the linguistic expressions and wording accuracy of students' answers will largely affect the final score, so this study focuses on the automatic determination of text semantics and language score points with fuzzy semantic similarity methods [21, 22]. The deep learning method is used to abstractly represent the deep semantic and linguistic features of the text. This study proposes a method to analyze and extract deep semantic features of text and shallow text features, then designs an automatic scoring model for the English translation, fuses the algorithm models, introduces an algorithm based on fuzzy semantic similarity for text retrieval, selects multiple fuzzy semantic similarities, calculates the final score by combining semantic features through regression or classification algorithms, forms an algorithm model for English translation scoring, and after model training, gets the optimal algorithm model that is obtained after model training, and then experimental validation is conducted. The word vectors trained on the monolingual corpus are uniformly mapped in the generic vector space to obtain the generic word vector embedding space. The model is trained using meta-learning, and a preliminary translation model, the initial model parameters, is obtained by training with the English bilingual training set and validation set, and then, the English bilingual test set is trained with the model parameters for fast adaptation, and a suitable translation model is finally obtained through training and fine-tuning [23]. At the same time, for the shortcomings of the nonautoregressive translation model, the knowledge distillation method is applied to it, which can significantly improve the English translation effect while enhancing the generation rate.

The article "Construction of English Translation Model Based on Neural Network Fuzzy Semantic Optimal Control" was published in 2022. Journal: Comput Intell Neurosci.

## 2. A Study on English Translation Model Based on Neural Network Fuzzy Semantic Optimal Control

### 2.1. Neural Network Fuzzy Semantic Optimal Control of Translation Features

The English words are sorted and filtered by the English dictionary, and the top n words with similar meanings to the English words are selected as the auxiliary quantities for updating the English word vector [24]. Finally, the English word vector is updated by the exact word vector generation algorithm, and the final exact representation of the English words is calculated, and then, the exact representation of the whole text is obtained. The above additional text information and the traditional model training word vector are combined to complete the pretraining of the precise word vector. That is, when using the traditional model for training, the contextual text information is used to guide the model to learn the emotional word features according to the sentiment polarity of the sentences in the corpus and the polarity of the self-labeled seed words. The precision word vector pretraining model and the word vector update algorithm are the two core points of the whole model. The accuracy of the former directly acts on the auxiliary amount of updating English word vectors, which has an indirect effect on the English word vector results; the latter plays a decisive role in the final generated English results. The neural network fuzzy semantic optimal control translation model mainly consists of three parts: pretrained exact word vector, English word sorting and screening, and exact word vector generation. The overall structure is shown in Figure 1. Redundant punctuation and incorrect grammatical formatting often appear in the grammaticalized text. In order to make it easier and more accurate for the model to learn text features, these redundant information needs to be filtered out, for example, breaking long sentences into short sentences, removing redundant symbols, and correcting misspellings. Formatted data can indirectly improve the training efficiency of the model.

The article "Construction of English Translation Model Based on Neural Network Fuzzy Semantic Optimal Control" was published in 2022. Journal: Comput Intell Neurosci.

The feature learning model consists of three components: context words and the information of the words that make up these words, the English polarity information of the sentences, and the English polarity information of the seed words. The word vector is trained by combining the context words and the information of the words that make up these words. The extended skip-gram model can better integrate the other two components. The skip-gram model aims to predict the context words of a given word and optimize the English language by maximizing the average log probability of equation (1), where *H* denotes the corpus, *h* denotes the words in *H*, and *E*(*h*) denotes the context words for *h* within the specified window.

(1) $$\begin{array}{c} G\left(X_{1}\right)=\sum_{h=1}^{H}\frac{\ln\left(F\left(E\left(h\right)\right)\right.}{2}|h. \end{array}$$

The English information of the sentences is added during the word vector training. This is performed by incorporating the English information of the sentence into the training model by predicting the English polarity of the sentence. The implementation of this process is similar to the first part, except that the prediction focus is no longer on the context of the word but on the English polarity of the whole sentence [25]. Each sentence is represented as a vector s at the time of implementation, and the vector s is the average of the word vectors that make up the words of the sentence. The sentences in the corpus used in this study are annotated with English polarity so that the information on the English polarity of the sentences can be used to improve the training quality of the model. This process aims to maximize the English function of the sentences. As shown in equation (2), *K* represents the corpus, *k* represents the sentences in the corpus, and *S*(*k*) denotes the English polarity of the sentences. The same negative sampling optimization method is still used as in the first part [26].

(2) $$\begin{array}{c} G\left(X_{2}\right)=\sum_{k=1}^{K}\frac{\ln\left(F\left(S\left(k\right)\right)\right.}{2}|k. \end{array}$$

During the training process, the English polarity of words is fully considered in conjunction with the acquired seed English dictionary, and more English information is incorporated into the word vector learning process by predicting the English polarity of words. The English polarity of which is divided into three categories: positive, negative, and other. The English of this process also maximizes the logarithm of English probability. As shown in equation (3), *A* denotes the seed lexicon, *S*(*k*) denotes English polarity, and *ν*^*ab*^ denotes the auxiliary vector. The other parameters have similar meanings to those in the above two parts of equation.

(3) $$\begin{array}{c} G\left(X_{3}\right)=\sum_{h,k=1}^{H,K}\frac{\ln\left(F\left(E\left(h\right)\right)\right.*F\left(S\left(k\right)\right)}{2}|h.k+\sum_{a,b=1}^{A,B}\log\left(\mu *\left(X_{a}^{b}*\nu^{ab}\right).\right. \end{array}$$

From the trained corpus lexicon, the top *k* words are selected in descending order of frequency, and the *k* words are manually labeled with English polarity [27]. The number of seed words is small, and the current word set needs to be extended to generate a more complete lexicon. Considering the hit rate and accuracy in seed word matching, the seed English lexicon should also contain the most common English words in the corpus to improve the training efficiency of the model and the final classification performance. Therefore, the initial selection of k high-frequency words from the original corpus, based on these words, and the use of synonym word forests to find words with semantic similarity to the high-frequency words can satisfy this extended requirement.

The article "Construction of English Translation Model Based on Neural Network Fuzzy Semantic Optimal Control" was published in 2022. Journal: Comput Intell Neurosci.

### 2.2. Construction of English Translation Model with Fuzzy Semantic Optimal Control

In ITS-UKF, several multistem fuzzy rules are established according to certain English translation features of English, and the antecedent parameters of these rules are fuzzy divisions of English translation features while the posterior parameters are English translation models of some English translation amounts established [28]. Similar to the traditional interactive multimodel, these rules can be transformed to interact with each other, and different fuzzy rules in ITS-UKF will transform to interact with each other by themselves according to the intersection degree of fuzzy affiliation function between fuzzy rules. The weight of each model in ITS-UKF and the antecedent parameters are formed into a knowledge system, and the neighborhood rough set is used to reduce and eliminate redundant models. At the same time, the excessive rough set reduction will consume a lot of computing power and lose effective information. According to each time and each model residual, an adaptive reduction judgment algorithm is proposed, which monitors the tracking situation through the residual, adaptively performs feature rereduction, and then simplifies the features.

It may not be set to *X*_*i*_^*j*^ that the fuzzy set of translated English being divided under the *j*th feature at the time *i*. The closer the fuzzy sets of different rules and their antecedent parameters are to each other, the higher the transfer change between rules. At the time *i*, the transfer probability of transforming fuzzy set *E* to fuzzy set *S* is shown in equation (4), where ∏(*E*, *k*) represents the intersection degree between fuzzy set *E* and fuzzy set *k*, *nJ* represents all fuzzy sets under the *j*th feature, and *E*, *k* ∈ *nJ*. The optimal control rule of neural network fuzzy semantics should be the hyperplane state value, and the general hyperplane FCM algorithm is not applicable. Here, the FCRM clustering algorithm is applied to realize the clustering of the overclocking surface data.

(4) $$\begin{array}{c} G\left(X_{i}^{j}=E|X_{i+1}^{j}=S\right)=\frac{\prod \left(E,k\right)}{\sum_{k=1}^{J}\prod \left(E,k\right)}. \end{array}$$

The model probability of prediction is calculated as shown in equation (5), in which *ω*_*h*+1_^*k*^ denotes the normalized probability of the *k*-th fuzzy rule at *h* + 1 moment. *ω*_*h|h*+1_^*k*^ denotes the mixing probability of total other fuzzy rules transformed to the *k*-th fuzzy rule.

(5) $$\begin{array}{c} \omega_{h|h+1}^{k}=\sum_{i=1}^{H}\varsigma \left(i,j\right)*\omega_{h+1}^{k}. \end{array}$$

The mixing probability is normalized as follows, as shown in equation (6), where *ω*_*h|h*+1_^*k|i*^ is the normalized mixing probability when the *i*-th fuzzy rule is transformed to the *h*-th fuzzy rule at the moment *h* + 1.

(6) $$\begin{array}{c} \omega_{h|h+1}^{k|i}=\sum_{i=1}^{H}\frac{\varsigma \left(i,j\right)*\omega_{h+1}^{k}}{\omega_{h+1}^{k}}. \end{array}$$

When the difference △ between the estimated result of a certain model and the observed result is large, it can be assumed that the English language at this time may not be translated into English by the English translation model that cannot describe the current English translation status, and it may begin to maneuver. In other words, a certain threshold can be set, and when the difference Δ between the predicted result of a certain model and the observed result is larger than this threshold, it means that the English may not be translated in this way English. This is applied to feature selection. First, the difference between the predicted observation *S*(*h*_*k*_^*i*^) and the observation *G*(*h*) is calculated for a set of all models at the current moment.

(7) $$\begin{array}{c} \Delta \omega \left(i\right)=\frac{1}{\sum_{h=1}^{S}\left(G\left(h\right)-S\left(h_{k}^{i}\right)\right.}, \end{array}$$

*F*(*ϕ*) is trained to predict the embedding vectors. Also, we choose cosine fuzzy semantic similarity as a neighboring metric for the semantic similarity between word vectors. The equation of the English function for training is equation (8). After the training of the model, we get *E*(*h*), with the help of which we can get the word vectors of unregistered words on the test set. In equation (8), *S*(*k*) is the input, and it is obtained using fuzzy semantic optimal control. The flowchart of fuzzy semantic optimal control is shown in Figure 2.

(8) $$\begin{array}{c} \phi =\sum_{\omega \left(i\right)}\sum_{\omega \left(h\right)}\sin\left(F\left(\phi \right)*E\left(h\right)*S\left(k\right),J\left(\omega \left(i\right)\right)\right). \end{array}$$

The article "Construction of English Translation Model Based on Neural Network Fuzzy Semantic Optimal Control" was published in 2022. Journal: Comput Intell Neurosci.

### 2.3. Evaluation of Neural Network Controlled English Translation Model Training

Usually, the word vectors used for semantically similar word pairs also have higher similarity, the calculated cosine similarity value will be higher and vice versa, and the dataset itself carries a manually labeled fuzzy semantic similarity value. Therefore, the semantic relevance of the word vectors can be measured by calculating Spearman's correlation coefficient between the actual cosine values and the artificially labeled values, where *i* denotes the number of word pairs and *h*_*i*_ denotes the difference between the corresponding ordinal numbers of the same word pairs in different sorting sequences after sorting the word pairs according to the calculated cosine and labeled values.

(9) $$\begin{array}{c} G\left(i\right)=\sum_{i=1}^{N}\frac{\sqrt{h_{i}^{2}}}{i*\left(i^{2}-1\right)}*100\%. \end{array}$$

When constructing the model, the shallow text features of word co-occurrence, text length, number of words in each lexical category, word list size, and deep semantic features were selected for the features of English text. Only representative shallow text features were selected, on the one hand, because the constructed scoring model focuses on using a deep neural network to do feature extraction, which contains features such as word meaning, word order, and sentence order, and is not repeatedly extracted, and on the other hand, to make the model applicable to English text. The linguistic shallow features mainly include two aspects of words and syntax. As shown in Table 1, the model mainly judges the pros and cons of answers based on similarity features and semantic features. For the semantic understanding of English-translated texts, especially in the case of diverse language expressions but the same semantics, it can score more accurately. At the same time, the understanding of polysemy and contextual relevance is also sufficient. In addition, the requirements for the size of the training set are not harsh. By calculating the weights through the attention mechanism, the influence of similarity features and semantic features on the final score can be adjusted.

The fuzzy semantic similarity of shallow linguistic features and the fuzzy semantic similarity of deep semantics are separately calculated, and the fuzzy semantic similarity is selected and combined with the deep semantic features to calculate the assigned weights to obtain the final score. The selection of the fuzzy semantic similarity method is explained in chapter 4. The existing English translation scoring models are mainly divided into two types of methods; the first one focuses on extracting shallow text features with a large number of dimensions and calculating the fuzzy semantic similarity with standard English translations; the second one treats scoring as a simple classification problem by representing the text by vectors or combining shallow text features and does not consider the influence of fuzzy semantic similarity with standard English translations. The limitations of these two types of methods are as follows: the first type of method is lacking for semantic extraction, which may lead to only lower scores when students' English translations are semantically identical to standard English translations but with special textual representations; the second type of method requires a large amount of training data, which may lead to lower scoring accuracy if the model is not sufficiently trained.

The article "Construction of English Translation Model Based on Neural Network Fuzzy Semantic Optimal Control" was published in 2022. Journal: Comput Intell Neurosci.

The neural network-controlled English translation model is mainly based on fuzzy semantic similarity features and semantic features to discriminate the merits of the English translation, and it can score more accurately for the semantic understanding of English translated texts, especially when the language expressions are diverse but semantically identical. It also has a more adequate understanding of polysemy and contextual association. It is not demanding on the size of the training set, and the size of the influence of fuzzy semantic similarity features and semantic features on the final score can be adjusted by the way of calculating weights through the attention mechanism.

Response generation uses neural networks to encode and decode the input text and knowledge. A neural network is a deep network that contains only attention mechanisms. He has the advantage of being able to process all words or symbols in a sequence in parallel while using self-attention mechanisms to combine context with more distant words, thus improving the disadvantage of slow training of RNN networks. By processing all words in parallel, each word is allowed to notice other words in the sentence in multiple processing steps. It can also increase to very deep depths to fully exploit the properties of deep neural network models and improve the accuracy of the models. The response generation part and the knowledge decision part are jointly trained together at the same time, and the model is trained in a process similar to multitask learning, while the reinforcement learning model is trained to learn how to make knowledgeable decisions, and the codec model learns how to generate responses based on input utterances, context, and selected knowledge. Through each round of interactive dialogues, the optimal path is found in the subgraph starting from the initial topic entity and finally stopping at the English topic entity. The reinforcement learning agent is trained to learn to find the optimal topic transfer path by using a sequence of topics with known initial and English topics and conversation pair data.

The article "Construction of English Translation Model Based on Neural Network Fuzzy Semantic Optimal Control" was published in 2022. Journal: Comput Intell Neurosci.

## 3. Analysis of Results

### 3.1. Analysis of Optimal Control Translation Algorithm

In the training process of the algorithm, a complete epoch process includes the updating of training parameters, testing, and validation of the algorithm. In the actual training process, the data need to be trained for several iterations to make the algorithm achieve the training effect of convergence fitting. In this experiment, different numbers of iterations are selected and the results are shown in Figure 3. From the above experimental results, we can see that the algorithm achieves the highest accuracy on the Data Hall dataset when the epoch is 7, and the algorithm achieves the highest accuracy on the NLP&CC2014 and ChnSentiCorp datasets when the epoch is 8. The algorithm achieves the highest accuracy on both NLP&CC2014 and ChnSentiCorp datasets when the epoch is 8. Therefore, the above experimental results show that the algorithm can obtain the best classification results in a short time by choosing the optimal number of iterations during training.

To verify the accuracy and effectiveness of the SA-RNN-CNN algorithm, we compare the three datasets used in this study with LSTM, BiLSTM, CNN, Self-Attention, and CNN-RNN algorithms. The CNN-RNN is an algorithm. The algorithm first obtains the phrase representation of the text using CNN, then obtains the sentence representation of the text as a whole using bidirectional RNN, and finally averages the sentence representation and achieves the classification by softmax classifier. The experimental results are shown in Figure 4. From the experimental results, it can be seen that the SA-RNN-CNN algorithm achieves the highest classification accuracy on all three datasets, while the BiLSTM algorithm achieves the lowest loss rate. The classification accuracies of the SA-RNN-CNN algorithm and CNN-RNN algorithm are close to each other, and the SA-RNN-CNN algorithm has 0.93%, 0.95%, and 1.03% higher accuracy and 0.4279, 0.4245, and 0.4085 lower loss rate than the CNN-RNN algorithm, respectively, which are much lower than the loss rate of CNN-RNN algorithm; BiLSTM algorithm achieves the lowest loss rate, but the SA-RNN-CNN algorithm is 5.18%, 5.95%, and 6.51% more accurate than the BiLSTM algorithm, and the loss rates are closer and 0.0213, 0.0378, and 0.0335 higher, respectively.

The article "Construction of English Translation Model Based on Neural Network Fuzzy Semantic Optimal Control" was published in 2022. Journal: Comput Intell Neurosci.

### 3.2. English Translation Model Performance Analysis

A comparison experiment was conducted to verify the effectiveness of NTM in English translation by evaluating the BLEU values and the time consumption distribution. After the experimental training, the trend of BLEU values of the three experimental models is shown in Figure 5. When the training reaches 100,000 steps, the model starts to enter the convergence stage, and the growth of the BLEU value starts to slow down, and when it reaches about 550,000 steps, the BLEU value of the model is stable and the best BLEU value of training is obtained. The best BLEU value of the three models is 65.48.

Figure 6 shows the trend of time consumption of the three experimental models. In Figure 6, it can be seen that the time consumed by the three groups of translation models gradually increases with the increase in the number of training steps, but the time consumed by the three groups of experiments remains at a lower level compared with the transformer model because the three groups of experiments adopt the English translation model based on the NAT architecture. According to the trend of the line change, we can understand that the English machine translation incorporating the NTM architecture does not greatly change in terms of time consumption, and the time consumption is slightly higher than that of the NAT + KD + MAMML translation model, which still maintains a lower level of time consumption. Based on the NAT architecture, fused NTM can effectively improve the quality of English neural machine translation. The NAT model that integrates the meta-learning strategy can further improve the performance of Mongolian-Chinese machine translation. Compared with the NAT model that only performs knowledge distillation processing, it finally improves the BLEU value by 2.3 points and improves 5.1 points of BLEU compared with the transformer model. The time consumption is much lower than the time consumed by the transformer model and slightly higher than the time consumed by the NAT + KD model.

The model is supplemented with contextual semantic information by the excellent storage capacity of the external memory of neural Turing machines to improve the translation effect. Then, we build an English translation model based on NTM and word-level attention mechanism, use external memory to write and read contextual semantic information, and set the relevant experimental parameters; next, we conduct group experiments on the built English translation model to verify the effectiveness of NTM in English translation. Finally, the experimental results are compared to verify the effectiveness of NTM on English machine translation based on NAT architecture, which can further improve the quality of English neural machine translation while maintaining the low time consumption of the model.

The article "Construction of English Translation Model Based on Neural Network Fuzzy Semantic Optimal Control" was published in 2022. Journal: Comput Intell Neurosci.

### 3.3. Simulation Analysis of English Translation Model Training

To test the effect of inheritance features on the model's ability to predict long-term returns, experiments are conducted on sentences of different lengths.  Figure 7 shows the performance of the tested model at different sentence lengths. It can be seen that the proposed model outperforms the benchmark model in almost all length intervals. In particular, when predicting long sentences, the proposed model can obtain better BLEU scores. Intuitively, the experimental results demonstrate that the DSF module can help the model achieve better long-term returns than local optima, and this difference is more obvious when the sentence length is longer. It can also be seen that the DSF-E2D model can perform generally better than the E2D-RL model when short sentences are used. We believe this is because the generation of short sentences is more dependent on the current per-word probability rather than on the long-term payoff. However, the E2D-RL model fine-tunes the model again after pretraining by maximizing the likelihood probability per word and the expected payoff, which makes the model effect more favorable to the prediction of long sentences to the detriment of short sentences. Unlike them, the proposed model calculates a 2-value for a group of similar words, and this value only slightly corrects the probability distribution of all words without destroying the pretrained model. Therefore, the proposed model performs better on short sentences relative to the E2D-RL model.

We briefly test the migration learning capability of the DSF-E2D model. The test is performed by replacing the evaluation method of the model when the training is close to convergence, i.e., replacing the BLEU value with the ROUGE value. The experimental results are recorded in Figure 8. An interesting phenomenon can be found that DSF-E2D can quickly adapt to the change in the evaluation method. It only needs to relearn the parameters *w* of the reward network to achieve a better evaluation score.

In this study, we use SF to unify the training and testing process in English and give the model the ability to focus on generating whole sentences. The proposed model shows significant improvement by training and testing on a large-scale bilingual corpus. We intend to apply this model to more text generation tasks in the future, especially dialogue systems, and use its inherited features to solve the problem of transfer learning of dialogue models trained on different domain corpora.

The article "Construction of English Translation Model Based on Neural Network Fuzzy Semantic Optimal Control" was published in 2022. Journal: Comput Intell Neurosci.

## 4. Conclusions

To address the lack of consistency in English translation models, this study considers English sentence features as the most important part to reflect consistency. Therefore, this study sets up some English translation-related information bases, retrieves information in the information bases through the attention mechanism, and then fuses the attention retrieval mechanism into the end-to-end generation model. The generation model compares the probability of generating words in the lexicon with the probability of generating information in the information base when generating words so that it can generate responses containing English information when English information-related questions need to be answered. Traceless Kalman maneuver English tracking algorithm is based on neural network fuzzy semantic multimodel. To address the problem that the set of models in traditional multimodel algorithms cannot cover all English translation models, the ITS-UKF algorithm uses the powerful fitting ability of neural network fuzzy models to select some English translation features of English as the system antecedents of neural network fuzzy models and fuzzy partition them to form several fuzzy rules. At the same time, each rule uses different traceless Kalman filtering algorithms to calculate the posterior of the neural network fuzzy model. Finally, the FCRM algorithm is iteratively used to compute the optimized updated preconditioner parameters. The simulation experiments demonstrate that ITS-UKF has better translation error performance compared with the traditional IMM algorithm. The experimental results verify the effectiveness and feasibility of this method. However, as the number of neural network layers increases, the computational complexity also increases, and it will be affected in terms of training time and speed. Meanwhile, since the research of optimal control-based neural machine translation is still in its infancy, most of the external tools for optimal control slicing are not mature enough. Therefore, the next step is to reduce the computational complexity of the model, improve the translation speed, and optimize the external optimal control slicing tools.

## Figures and Tables

**Figure 1:** Neural network fuzzy semantic optimal control translation model.

The article "Construction of English Translation Model Based on Neural Network Fuzzy Semantic Optimal Control" was published in 2022. Journal: Comput Intell Neurosci.

**Figure 2:** Fuzzy semantic optimal control flowchart.

**Figure 3:** Line graph of the relationship between the number of iterations of the algorithm and the variation of the loss rate.

**Figure 4:** Classification accuracy and loss rate of different algorithms on each dataset.

**Figure 5:** The trend of BLEU value in 5 groups of experimental models.

**Figure 6:** The trend of consumption time of three groups of experimental models.

**Figure 7:** BLEU scores of the model on different sentence lengths in English translation.

**Figure 8:** Performance of DSF-E2D model and E2D-BS model after changing evaluation criteria.

**Table 1:** Attributes of superficial language features.

Serial number	Characteristics of words	Features of sentences
1	Number of words (text length)	English translation structure
2	The proportion of words by part of speech	Almost average sentence length
3	Vocabulary size	The number of words in each part of speech

## Data Availability

The data used to support the findings of this study are available from the corresponding author upon request.
